The article "Chaperone-mediated autophagy: roles in neurodegeneration" was published in 2014. Journal: Transl Neurodegener.

# Chaperone-mediated autophagy: roles in neurodegeneration

**DOI:** 10.1186/2047-9158-3-20

**Published:** 2014-09-21

**Authors:** Gang Wang, Zixu Mao

**Affiliations:** 1 Departments of Pharmacology and Neurology, Emory University School of Medicine, Atlanta, GA 30322, USA; 2 Center for Neurodegenerative Diseases, Emory University School of Medicine, Atlanta, GA 30322, USA

**Keywords:** Chaperone-mediated autophagy, Protein posttranslational modifications, Neurodegeneration, Alzheimer’s disease, Parkinson’s disease

## Abstract

Chaperone-mediated autophagy (CMA) selectively delivers cytosolic proteins with an exposed CMA-targeting motif to lysosomes for degradation and plays an important role in protein quality control and cellular homeostasis. A growing body of evidence supports the hypothesis that CMA dysfunction may be involved in the pathogenic process of neurodegenerative diseases. Both down-regulation and compensatory up-regulation in CMA activities have been observed in association with neurodegenerative conditions. Recent studies have revealed several new mechanisms by which CMA function may be involved in the regulation of factors critical for neuronal viability and homeostasis. Here, we summarize these recent advances in the understanding of the relationship between CMA dysfunction and neurodegeneration and discuss the therapeutic potential of targeting CMA in the treatment of neurodegenerative diseases.

## Introduction

Based on delivery mechanisms of cargo destined for the lysosomes, autophagy can be classified into three types, macroautophagy, microautophagy, and chaperone-mediated autophagy (CMA) [1]. CMA selectively delivers cytosolic proteins with a CMA targeting motif to lysosomes for degradation and plays an important role in protein quality control (QC) in cells [2-4]. Recently, a growing body of evidence supports that dysfunction of CMA may contribute to the etiologic and pathogenic process of neurodegenerative disease. Here, we describe recent advances in the understanding of the relationship between CMA dysfunction and neurodegeneration.

## CMA: a unique machinery for cellular homeostasis

### Basic components of CMA machinery

At the cellular level, CMA is a vital multi-step process. It involves recognition of potential substrates by the chaperone protein, heat shock cognate protein 70 (Hsc70), delivery of substrates to lysosomes, transport of unfolded substrates into lysosomes by receptor LAMP2A, and degradation (Figure 1).

**Figure 1:** **Steps and regulation of CMA.** “X” represents local region or site of regulation.

### Substrate-CMA motif protein

Generally, a typical CMA substrate protein contains a KFERQ-like motif in its sequence which can be recognized by the chaperone protein Hsc70 when exposed and not buried in a protein fold. Two characteristics associated with this motif are notable: (1) motif plasticity: previous analysis established that about 30% of cytosolic proteins contain the putative KFERQ motif in their primary sequences [5]. Recent studies found that post-translational modifications (PTMs) such as phosphorylation and acetylation can change amino acid charge and can turn an atypical motif which differs by one residue from the standard one into a more effective motif recognizable by the CMA process [6-8]. Alternatively, a string of imperfect and overlapping motifs can also serve to mediate the CMA process [9]. Additionally, some of the KFERQ motifs in their native conditions may be concealed by normal protein folding in the interior of a protein, which is thought to prevent degradation via CMA under normal, unstressed conditions. After misfolding, partial unfolding, or PTMs that may influence the recognition motif directly or allosterically, conformational changes allow CMA substrate motifs to be exposed and the respective proteins then become suitable CMA cargo [3,10]; (2) multiple compartment sources of substrate proteins: prior studies suggested that soluble cytosolic proteins could be degraded by CMA [11,12]. But any proteins which can be delivered to the cytosol from other compartments via cellular trafficking may be regulated by CMA. These include plasma membrane proteins, organelle membrane proteins, or nuclear proteins [2,13]. Furthermore, it is theoretically possible that cleaved protein fragments under various conditions can also be degraded by CMA as long as they retain a CMA recognition motif.

### Ambiguous chaperone-Hsc70

The cytosolic Hsc70 (cyt-Hsc70) is a multifunctional chaperone involved in different cellular functions, including protein refolding and targeting to different organelles [14,15]. For CMA, cyt-Hsc70 protein interacts with substrate proteins via their CMA recognition motifs to deliver CMA substrates to lysosomes for degradation. In addition to lysosomes, Hsc70 can also deliver proteins with a CMA motif to late endosomes where they undergo degradation through endosomal microautophagy (e-MI) [16]. However, the mechanisms that determine to where the target proteins are delivered (CMA or e-MI) are not clear and remain to be elucidated. A recent study has shown that Hsc70 can bind to protein aggregates and target them to lysosomes via chaperone-assisted selective autophagy (CASA) [17]. Therefore, CMA is just one of the tasks performed by Hsc70.

In addition to cyt-Hsc70, lysosome-associated Hsc70 (lys-Hsc70) localized within the lumen of lysosomes is also involved in CMA [18]. Blockage of epitopes on lys-Hsc70 interrupts the internalization rather than membrane binding of CMA substrate proteins. Hence, lys-Hsc70 plays a key role in substrate translocation after delivery to lysosomal surface by cyt-Hsc70. Under oxidative stress or starvation, both the amount of lys-Hsc70 in lysosomes and the number of lysosomes with lys-Hsc70 increase remarkably [10,19]. But whether and how pathological conditions alter lys-Hsc70 remains unclear.

### CMA receptor-LAMP2A

The lysosome-associated membrane protein type 2a (LAMP2A), in contrast to the other two splice variants, LAMP2B and C, is the receptor for CMA substrates. The LAMP2A-mediated translocation step is rate limiting for the whole CMA process [20]. CMA substrate protein binds to the c-terminal cytosolic tail of LAMP2A at the lysosomal membrane and this interaction quickly promotes the monomeric form of LAMP2A to assemble into a high molecular weight complex of about 700 Kd [20,21]. Once a substrate has been released into the lysosomal lumen, the complex dissociates into monomers again. In fact, binding of substrate proteins is restricted to monomers of LAMP2A. In contrast, translocation begins only after multimerization of LAMP2A. Interestingly, Eskelinen and co-workers found that LAMP-1 and -2 double deficiencies did not affect CMA-mediated proteolysis in mouse embryonic fibroblasts, suggesting that LAMP2A may not be the only receptor for CMA and that there are likely alternative receptor mechanisms for the CMA process [22].

### Lysosomes: an advanced organelle

Lysosomes are ubiquitous membrane-bound intracellular organelles involved in many cellular processes and considered to be a crucial regulator of cellular homeostasis rather than waste bags [23]. As the destination for CMA, lysosomes maintain a highly acidic pH within their lumen in order to digest delivered contents and then to drive efflux of digested metabolites, thereby recycling key digested components. The function of lysosomes is critically dependent on both soluble lysosomal hydrolases (e.g. proteases, lipases, glycosidases and nucleases) and lysosomal membrane proteins (e.g. lysosome-associated membrane proteins) [24,25].

Recent research has revealed that the transcription factor EB (TFEB) can enter the nucleus and bind to coordinated lysosomal expression and regulatory (CLEAR) elements, and induce the transcription of genes involved in lysosomal biogenesis [26,27], acting as a master regulator of lysosomal function to coordinate the activity of the lysosomal network in response to changing environment and cellular needs [28,29]. The pathways that mediate the fate of the end products of lysosomal digestion are poorly understood. Generally, the metabolites of lysosomes, degradation end products, will be reused for protein synthesis or cellular respiration in the cytosol after lysosomal efflux via diffusion or transport through specific transporters (lysosomal membrane proteins that export lysosomal degradation products) [30-32]. However, the detailed mechanisms that maintain the balance between degradation and recycling processes require further investigation (Figure 1).

### Regulatory mechanisms of CMA

Although the basic steps of the CMA process are well characterized, our understanding of how CMA is regulated is very limited. The levels of CMA activity are believed to change constantly, allowing adaptation to both immediate and long-term needs of the cells. Some known regulatory mechanisms include the following:

(1) Regulation at a molecular level: CMA activity could be regulated by modulating substrate binding via LAMP2A and also substrate translocation via lys-Hsc70.

Changes in LAMP2A abundance due to changes in its synthesis, degradation, redistribution, and conformation at the lysosomal membrane have profound effects on CMA activity and flux [21]. Additionally, the stability of the CMA translocation complex of LAMP2A has been found to be modulated by a GFAP-EF1a complex [33]. For lys-Hsc70, an increase in its level may lead to a gradual augmentation of CMA activity. These mechanisms have been reviewed in detail elsewhere [15,19,34-36].

(2) Regulation at a pathway level: CMA activity could be regulated by modulating the equilibrium of flux through the autophagic/proteolytic system, and the equilibrium of influx and efflux across the lysosomal membrane.

In cells, a proteostasis network comprised of CMA, macrophagy (MA), and the ubiquitin-proteosome system (UPS) exists [37]. For cellular protein and metabolite homeostatsis, an intricate and delicate equilibrium among these pathways needs to be maintained. Alteration of any single pathway will precipitate changes in the other proteolytic pathways. For example, CMA blockage could induce MA up-regulation. On the other hand, blockage of MA results in CMA activation [38,39]. Similarly, a decrease in CMA or MA activity has been found to lead to changes in the activity of the UPS [40,41]. The molecular mechanisms underlying the cross-talk among these different pathways have not been fully elucidated. Yet, there is some experimental evidence to suggest that this may also involve lys-Hsc70 and/or LAMP2A [42]. The equilibrium of influx and efflux transport across the lysosomal membrane is poorly understood [30]. Processing a subset of soluble cytosolic proteins by CMA will lead to the generation of a group of degradation end products for reuse. If the end products are in shortage or excess for subsequent synthesis of essential proteins, there should be compensatory alterations in the influx and efflux processes. Some studies have revealed that a putative amino acid efflux transporter in lysosomes, Atg22, plays a role in autophagy. Atg22 cooperates with two other proteins, Avt3 and Avt4, in supporting amino acid transport [43]. However, whether Atg22 participates in the regulation of CMA is unknown and this and other factors that could affect the final steps of CMA clearly require further investigation.

### The roles of CMA in neurodegeneration

Given the important role of CMA in maintaining cellular homeostasis, it is not surprising that CMA dysfunction has been linked to the pathogenic processes of severe human disorders. Because of their postmitotic nature, neurons are especially sensitive to homeostatic changes. Both down-regulation and compensatory up-regulation of CMA activity have been shown to be associated with neurodegeneration [7,44,45]. Interestingly, among these studies, increasing CMA activity has only been reported in relatively younger HD mice rather than older mice, suggesting that there may be heterogenous alterations of CMA between early and late stages of a pathogenic process [45].

### Effects on CMA by risk factors associated with neurodegeneration

Certain environmental elements, genetic variations, and aging have all been identified as etiological factors associated with various neurodegenerative diseases [46,47]. The potential role of CMA dysfunction in neurodegenerative disease is a subject of increasing interest. This has led to some efforts aimed at addressing the relationship between CMA and other known etiological factors.

(1) Environmental risk factors: compared to our understanding of how toxins dysregulate MA machinery, little mechanistic detail is known about the interaction between environmental factors and CMA. Of the few studies focusing on the effects of neurotoxins on CMA activity, Marin and co-workers showed that the levels of LAMP2A and Hsp90 are increased in the nigral region in the 6-hyroxydopamine (6-OHDA)-induced unilateral lesion rat model, providing *in vivo* evidence for toxin-induced change in CMA activity [48]. Consistently, a recent study by Gao et al. found that 6-OHDA induces an increase in LAMP2A in the substantia nigra pars compacta of mouse brain [43]. In cellular models where experimental conditions can be more precisely controlled, it has been shown that limited exposure to moderate levels of insults (toxin or stress) leads to an increase in CMA [43,49]. This appears to represent a cellular protective response to alleviate toxin-induced damage. But persistent exposure to high levels of toxic insults has been clearly demonstrated to result in a severe decrease in CMA activity. However, the effects of these various toxins on CMA substrates are complex and may not always be related directly to CMA. For example, Sala and colleagues reported that the mitochondrial toxin rotenone induces an increase in the levels of CMA substrates synuclein and MEF2D [50]. But the changes in these protein levels appeared to be due to changes in the regulation of their de novo synthesis rather than inhibition of their CMA-mediated degradation.

(2) Genetic risk factors: the mutant variants of several pathogenic proteins bearing CMA-targeting motif(s) have been shown to impair CMA activity. These include α-synuclein, ubiquitin C-terminal hydrolase L1 (UCH-L1), and leucine-rich repeat kinase 2 (LRRK2) [51-53]. Aside from being more resistant to CMA degradation, an emerging common mode of action for several of these pathogenic variants is that they exert negative effects on CMA via inhibiting the CMA process at the lysosomal membrane and interfering with the degradation of other CMA substrates. In addition, our previous study identified that high levels of either wild type or PD associated α-synuclein mutant disrupt CMA-mediated regulation of neuronal survival factor, MEF2D, which plays a role in neuronal stress and death [9].

(3) Aging: Studies of aged rodents and humans have revealed that aging is associated with a decline in CMA activity. This impairment of CMA in aging is mainly due to a decrease in the levels of LAMP2A at the lysosomal membrane secondary to its reduced stability instead of decreased de novo synthesis of this critical CMA receptor [54].

## CMA substrate proteins and pathogenic roles in neurodegenerative diseases

### CMA defects implicated in the etiology of neurodegenerative diseases

Accumulation of pathogenic CMA substrate proteins such as α-synuclein, in the form of insoluble inclusions, is a common hallmark underlying the degenerative process of many diseases, such as Parkinson’s disease (PD) and certain tauopathies. CMA can only degrade the soluble forms of these proteins. Once forming insoluble inclusions, they are much more resistant to CMA-mediated degradation. These aggregates may often exert a “clogging or blockage effect” at the lysosomal membrane, thus becoming toxic by inhibiting the CMA-mediated degradation of other cytosolic substrate proteins [51,55]. Although it is not clear whether CMA dysfunction may contribute to the initial formation of insoluble inclusions, it is quite possible that the “blockage effect” on CMA may exacerbate the formation of inclusion bodies by increasing misfolded protein concentrations in the cytoplasm. Despite this common “blockage” mode of action, the CMA dysfunction phenotype of different neurodegenerative diseases may not be completely identical since the expression levels of CMA markers, LAMP2A and Hsc70, and CMA activity itself, vary among different diseases. For example, CMA activity appeared to be up-regulated in HD in one study [45], and therefore, the increasing CMA activity may be a compensatory mechanism to promote clearance of Htt by CMA [56]. In contrast, a decrease in CMA activity has been reported in other neurodegenerative diseases, including PD and AD [44,57]. But even among this group of diseases, there may be differences in changes occurring along the CMA pathway. Alvarez-Erviti et al. found that the expression levels of LAMP2A and Hsc70 are significantly reduced in the substantia nigra pars compacta and amygdala of PD brains compared with age-matched AD and control brain samples [44].

### Pathogenic variants of CMA substrate protein in neurodegenerative diseases

Currently, several proteins involved in neurodegenerative diseases have been reported as CMA substrates (Table 1). The reported effects of these mutant variants on CMA functions are summarized therein. There is no doubt that the list of CMA-related pathogenic proteins will grow with future research.

**Table 1:** Pathogenic variants of CMA substrate protein in neurodegenerative disease

**CMA substrate/binding Protein**	**Physiology function**	**Pathogenic mutant variants**	**Molecular mechanism**	**Effects on CMA activity**	**Disease**
Ubiquitin C-terminal hydrolase L1 (UCH-L1) [52,58]	Neuronal deubiquitinating enzyme	I93M	Abnormal binding to LAMP2A to block degradation by CMA substrates	↓	PD
α-synuclein [51,55]	Function is not well understood	A30P, A53T	Abnormally high affinity binding to LAMP2A to prevent the translocation across the lysosomal membrane	↓	PD
Leucine-rich repeat kinase 2 (LRRK2) [59,60]	Involved in mitogen-activated protein kinase, protein translation control, programmed cell death, and activity in cytoskeleton dynamics	G2019S	Interference with the organization of the CMA translocation complex and cause defective CMA	↓	PD
Tau [53,57]	Stabilization of microtubules	FTDP-17 mutation (TauRDΔK280)	Oligomerization at the surface of lysosomes to disrupt the membrane integrity and blockage of normal CMA function	↓	AD
Regulator of calcineurin 1 (RCAN1) [61]	A mediator of stress- and Aβ-induced neuronal death	\	Mechanistic effects on lysosome unclear	↓	AD
Huntingtin [7,45,56]	Unclear and essential for development	Expansion of polyglutamine	Increased clearance via regulation of LAMP2A and lys-Hsc70	↑(early stages); ↓(late stages)	HD

Note: \ (No reports are currently available); ↓ (Decrease); ↑ (Increase).

### Summary and perspective

In summary, the identification of selective degradation of proteins relevant to neuronal survival and stress via CMA has expanded the repertoire of cellular mechanisms by which CMA may be involved in the pathogenesis of neurodegeneration. The methods currently available to study CMA allow for measurement of the steps of the entire CMA process and flux through these steps [62,63]. Combination of different types of approaches, including genetic method and CMA-modulating drug, should be useful to reveal additional mechanisms by which CMA dysfunction may trigger pathogenesis and enable the dissection of the specific steps of CMA which are dysfunctional in the pathogenic process. Agents capable of modulating lysosomal activity, for example, neutralizers of lysosomal pH like chloroquine, are currently tested in anti-cancer clinical trials [64,65]. Interventions to prevent CMA blockage and improve CMA throughput, particularly in the brain, may have therapeutic value in the treatment of neurodegenerative diseases and are therefore worth evaluating. In addition, a recent study has revealed a decrease in the level of Hsc70 in lymphomonocytes isolated from PD patients, suggesting that CMA associated proteins and/or cargoes may be explored as new biomarker(s) for neurodegeneration [66].

## Competing interests

The authors declare that they have no competing interests.

## Authors’ contributions

GW drafted and ZM critically revised the manuscript. Both authors read and approved the final manuscript.
